# Calbindin S100A16 Promotes Renal Cell Carcinoma Progression and Angiogenesis via the VEGF/VEGFR2 Signaling Pathway

**DOI:** 10.1155/2022/5602011

**Published:** 2022-09-15

**Authors:** Ning Wang, Rongjiang Wang, Jianer Tang, Jianguo Gao, Zhihai Fang, Meng Zhang, Xufeng Shen, Lingqun Lu, Yu Chen

**Affiliations:** ^1^Department of Urology, The First Affiliated Hospital of Huzhou Teachers College, Huzhou 313000, China; ^2^Zhejiang Academy of Medical Sciences, Hangzhou 310000, China

## Abstract

**Purpose:**

Recent research has indicated that the calcium-binding protein S100A16 promotes carcinogenesis and tumor growth in several forms of cancer. The objective of this study was to examine the relationship between S100A16 and renal cell cancer.

**Methods:**

By using The Cancer Genome Atlas (TCGA) database, the differentially expressed gene S100A16 was identified, and its appearance and link to the prognosis of persons with renal cancer were confirmed. Cox regression was used in multivariate analysis, and a nomogram was developed for internal validation. The correlation between S100A16 and immune cells was analyzed in the TIMER database. Moreover, the potential mechanism of action was investigated utilizing GO and KEGG enrichment analyses. Proliferation, migration, and angiogenesis were investigated in vitro, and the involvement of S100A16 in the undesirable biological events of renal cell carcinoma (RCC) was further explored.

**Results:**

S100A16 was the differentially expressed molecule identified through database screening. Malignant tissues showed higher S100A16 expression than noncancerous tissues, and S100A16 expression was mostly localized in the cytoplasm. According to the TCGA and KM-plotter datasets, patients with RCC and low S100A16 expression had superior OS, PFI, and DSS. The C-index of the nomogram was 0.754 (0.726–0.782), and the accuracy of the prediction model was high. The TIMER database shows that the expression of S100A16 is associated with immune infiltration and may play an important role in promoting tumor cell immune escape in the RCC tumor microenvironment. S100A16 may influence the biological processes of RCC via the VEGF/VEGFR2 signaling route and PI3K-Akt signaling pathway and through P53 alteration and cell cycle according to the gene enrichment technique. In vitro cytological experiments demonstrated that S100A16 knockdown can inhibit the proliferation and migration of renal cancer cells and the expression levels of VEGF, VEGFR2, and phosphorylated AKT within renal cancer cells, thereby inhibiting angiogenesis in renal cancer cells and resulting in a poor prognosis of RCC.

**Conclusion:**

A decrease in S100A16 expression may dramatically increase the OS, PFI, and DSS of patients with RCC and may thus be used as a biomarker for predicting RCC. It may be associated with the immune infiltration of RCC and play a crucial role in the immune evasion of tumor cells within the RCC microenvironment. Intervention of s100a16 can promote the progression and angiogenesis of renal cell carcinoma through the VEGF/VEGFR2 signal transduction pathway and lead to poor prognosis of renal cell carcinoma. These findings suggest a potential target for the development of anticancer strategies for renal cancer.

## 1. Introduction

Renal cell carcinoma (RCC) remains one of the most widespread tumors of the urinary system, after renal cylindrical epithelial cubicles. It accounts for approximately 4% of malignant tumors of the urinary system, and its incidence continues by approximately 3% annually. In 2018, a total of 400 000 persons were diagnosed with RCC globally [1]. The histological forms of RCC include pure cubicle carcinoma (70%), papillary compartment carcinoma (10%–15%), and chromophobe carcinoma (5%) [2]. The progression of renal cubicle carcinoma is subtle. Identifying patients with hematuria and belly figure remained identified. However, most of the patients have no obvious symptoms, and they are occasionally found in imaging examination during physical examination. Therefore, when diagnosed with RCC, most patients have dismal prognoses. Patients in the advanced stage have a mortality rate of less than 10% [3], and the effectiveness of treatments for RCC, including surgery, chemoradiotherapy, and endocrine therapy, is still inadequate [4]. In the early stages of RCC, surgical resection is curable. Approximately 25%–30% of patients had distant metastasis at the time of diagnosis, and 40% of patients return after surgical resection [5]. Radiotherapy and chemotherapy are ineffective against metastatic and recurring renal cell carcinoma, and options for tailored treatment are limited [6, 7]. Exploring biomarkers related to the onset and advancement of renal cell carcinoma may enhance future therapy methods and prognosis for RCC.

An S100 protein has 25 components. Each member is encoded by a separate gene [8]. The S100 protein family consists of acidic calmodulin proteins with low molecular weights [9], and each has two Ca^2+^-regulated EF-hand-type domains. The C-terminus is a common feature of all EF-hand proteins, and the S100 family members have extra N-terminal stands. The C-terminal EF-hand region is followed by a stretch of amino acids known as the C-terminal extension The area between the dual domains of the EF hand is known as the pivot. Among the different proteins, the variability of the C-terminal extension and hinge region was the greatest; hence, they dictate the protein's distinct biological features [10].

By interacting with target proteins, the S100 protein participates in biological events, including cell growth, differentiation, motility, contraction, transcription, gesture transmission, protein phosphorylation, cubicle survival, apoptosis, and cubicle round control [11]. Inflammation, neurological disorders, depression, dejected syndrome, cystic fibrosis, and tumor are linked to the S100 protein. S100A16, an S100 protein, located in the 1q21 region of human chromosome, was isolated from astrocytoma. S100A16 is widely expressed in specific tissue types such as adipose tissue and brain [12]. Additionally, S100A16 is strongly associated with the prognoses of several tumors. Tanaka et al. [13] showed that S100A14 and S100A16 interact with cytoskeleton dynamics and increase the invasiveness of breast cancer cells. Fang et al. [14] hypothesized that S100A16 promotes the growth and spread of pancreatic tumor via FGF19-mediated AKT and ERK1/2 pathways. In human prostate cancer [15], S100A16 promotes cell proliferation and metastasis through Akt and ERK cell signaling pathways. Through the JNK/p38 MAPK pathway, S100A16 inhibits the proliferation, migration, and invasion of colorectal tumor cells [16]. To date, no research has reported the prognoses of individuals with S100A16 and renal cell cancer.

Our research focused on the expression of S100A16 and its role in predicting the survival rate of renal cell carcinoma patients. In addition, bioinformatics analyses and in vitro tests were conducted to study the influence of S100A16 on the behaviour and underlying processes of tumor cells.

## 2. Materials and Methods

### 2.1. Data Analysis Using the TCGA Database

To examine the role of S100A16 in RCC, we analyzed data from the TCGA database (https://tcga-data.nci.nih.gov/).

### 2.2. Relationship between S100A16 and the Clinical Parameters of Patients with RCC in the TCGA Database

We obtained the clinical parameters of patients with RCC from the TCGA database and then analyzed the correlations among S100A16, these clinical parameters, and prognosis.

### 2.3. Construction and Evaluation of Nomograms

We generated nomograms according to the multivariable analysis results to estimate survival probabilities at 1, 3, and 5 years. The RMS R program was used in constructing nomograms including clinical characteristics related to S100A16 and calibration plots. Calibration and discrimination are the most often used approaches for assessing model performance. In this study, the calibration curve was graphically evaluated by mapping the nomogram prediction probability to the observed ratio, *t*, and the 45 degree line represents the best prediction value. Concordance index (C-index) was used in evaluating the discriminative power of the nomogram and was computed using a bootstrapping technique with 1000 resamples. It was also used in predicting the exactness of the nomograms and specific prognostic variables.

### 2.4. Relationship between S100A16 and Safe Cells in the TIMER Database

We constructed a bar graph from the TIMER record (https://cistrome.shinyapps.io/timer/) to display connection among S100A16 countenance and various safe cells in RCC.

### 2.5. GSEA Enrichment Analysis

Using Metascape (https://metascape.org/gp/index.html “*l*”/main/step1), a functional study was conducted online. Meta cape was augmented with distinct genes for functional analysis.

### 2.6. RCC Cell Culture

A hominoid croc cubicle stroke Caki-1 (obtained from ATCC, Manassas, VA, USA) was used. The cells were cultured in RMPI-1640 media (Thermo Fisher Scientific, MA, USA) supplemented with 10% fetal bovine serum (Thermo Fisher Scientific Inc., MA, USA). Two sets of Caki-1 cells were created: regulator cluster and sh-S100A16 groups. The media were changed as required, and cell cultures were maintained at 37°C in a humidified environment containing 5% CO_2_.

### 2.7. Reverse Transcription-Quantitative PCR Method to Detect mRNA Encoding S100A16

Approximately 100 mg of tumor and noncancerous flesh samples were collected from each participant. The tissues were ground into powder with liquid nitrogen, and 1 ml of TRIzol lysis solution was added. RNA was cut and reverse-transcribed into cDNA. Fluorescence quantitative PCR was performed using a fluorescence quantitative PCR apparatus. By using the 2-Ct technique, the quality of the mRNA of a target molecule was determined. S100A16 was found to be expressed in cancer and neighboring cancer cells.

### 2.8. In Vitro Cytological Experimental Verification

#### 2.8.1. Western Blot

After two times of washing with 4°C PBS, the cells were lysed in a cold RIPA buffer comprising proteinase inhibitors. Protein concentrations were measured with a BCA protein assess kit (Pierce, Rockford, IL, USA), and whole protein was denatured with 10% SDS-PAGE and transferred to a nitrocellulose membrane. The membrane was blocked with 5% skim milk in Tris-buffered saline containing 0.1% Tween-20 (tbst) for 1 hour at room temperature. The membrane was then treated immediately at 4°C with a primary antibody. After three times of washing with TBST, the films were gestated by a secondary antibody (anti-rabbit IgG) at room temperature and incubated for one hour. The film was washed with TBST three times, and an ECL reagent was used in identifying a target protein (EMD Millipore, MA, USA).

#### 2.8.2. Endothelial Cell Tube Formation Assay

For 24 h, Caki-1 cells were cultured in serum-free RPMI-1640 media for the preparation of a cell-conditioned medium. Then, 5000 HUVECs were plated on Slide Angiogenesis (Grafelfing, Germany) coated with Matrigel (BD science, New Jersey, United States) and treated with Caki-1-cell-trained media. Tube creation was photographed under a microscope, and the number of branches was determined.

#### 2.8.3. Apoptosis Assay

Cells were extracted and centrifuged at 1000 g*g* for 5 min for apoptosis examination. After the supernatant was removed, the cells were counted and resuspended in PBS. Reagents were added according to the protocol of the annexin/PI Kit (Beyotime, Shanghai, China). After incubation for 10–20 min at room temperature (20–25°C) in the dark, cells were collected and detected by FACS canto II (BD Sciences, New Jersey, USA).

#### 2.8.4. Statistical Analysis

Numerical study and visualization were performed using R (version 3.6.3). Equerry bundle (version 2.54.1) was used in downloading, and Limma bundle (version 3.42.2) was used in analyzing differences. GSEA was used in investigating the potential biological processes of S100A16. Survival was determined with the Kaplan–Meier method, and significance was tested. Spearman's correlation coefficient was used in determining correlations. A *p* value of 0.05 indicated statistically significant difference.

## 3. Result

### 3.1. S100A16 Expression Is Elevated in RCC

First, we performed renal clear cell carcinoma analysis with the TCGA database. We found that S100A16 was highly expressed in the majority of tumor tissues (Figure 1(a)). Additional analysis revealed that the expression of S100A16 was elevated in RCC tumor tissues (Figures 1(b) and 1(c)). The ROC curve revealed that the AUC for S100A16 was 0.779%, indicating that it had excellent predictive effect (Figure 1(d)).

In contrast to the clinical data of RCC patients, the expression of S100A16 was greater in RCC patients with advanced TNM stage. This result was consistent with prior TCGA results, indicating that S100A16 functions as an oncogene (Figure 2).

### 3.2. Correlation between S100A16 and RCC Prognosis in the TCGA Database

From clinical data of RCC in the TCGA database, we determined the effect of varying S100A16 expression. Patients with RCC and high S100A16 expression showed lower OS, DSS, and PF than those with low S100A16 expression (Figure 3(a)). Subgroup stratification analysis findings revealed that the prognoses of patients with RCC and low S100A16 expression were better (Figure 3(b)).

### 3.3. Nomogram Construction

Using the multivariable study results, we created a nomogram to predict 1-, 3-, and 5-year survival rates of patients with RCC. The nomogram C-index was 0.754 (0.726–0.782), and the prediction accuracy of the model was satisfactory (Figure 4(a)). Bias correction line is nearby to model bend (i.e., the 45-degree line) in the calibration plot, indicating good agreement between forecasted and observed values (Figure 4(b)).

We derived bar graphs to illustrate the relationship between S100A16 expression and diverse immune cells in RCC. Sort1 is favorably linked with the majority of invading immune cells, such as Th2, NK CD56 bright, DC, Tgd, pDC, NK, Th1, and mast cells. However, it was adversely related to the expression of *T* helper cells, Th17, and Tcm (Figure 5(a)). To evaluate the effect of S100A16 expression on the tumor microenvironment, we analyzed connection among S100A16 and specific immune cells. The results showed that S100A16 was strongly associated with the invasion of Th2, Th1, Tgd, TFH, pDC, and NK cells and negatively correlated with the invasion of Th17, Tcm, and *T* helper cells (Figure 5(b)). Subsequent research indicated that S100A16 was strongly linked to immune checkpoint-related markers CTLA-4, CD274, and PDCD1 (Figures 5 and 5(c)). These results provided valuable insights into the relationship between S100A16 and immune infiltration and showed that S100A16 may promote the immune evasion of tumor cells in the RCC tumor microenvironment, providing a reference for future fundamental research.

### 3.4. Correlation between S100A16 and Molecular Targeted Therapy Using Drug Target Molecules in the TCGA Database

Owing to the insensitivity of metastatic and recurring RCC to radiation and chemotherapy, comprehensive targeted therapy remains mostly used for treating late-stage disease. Sunitinib, bevacizumab, and erlotinib are recommended as first-line therapies, and sorafenib as second-line medication. Pazopanib, axitinib, and cabozantinib may be utilized as first- and second-line therapies for patients with RCC, depending on their individual circumstances. S100A16 demonstrated a positive association with AXL, EGFR, FLT3, KIT, MET, NTRK2, RET, TEK, and VEGFA, as shown by correlation research (Figure 6).

We conducted KEGG functional analysis using the Metascape online. By contributing within the VEGF/VEGFR2 signaling route, P53 alterations, cell cycle, and PI3K–Akt signaling system, S100A16 may influence the biological processes of RCC, resulting in varied prognoses. On the basis of these predictions, we hypothesized that the calcium-binding protein S100A16 may increase the growth and angiogenesis of RCC through the VEGF/VEGFR2 signaling pathway. This finding serves as a reference for our basic experimental investigation (Figure 7).

Gene biology biological process gene set from MSigDB was used. A total of 2000 random example permutations were conducted: FDR-q, false discovery rate; NES, normalized enrichment score; NOM-p, nominal *p* value.

### 3.5. S100A16 is Highly Expressed in Renal Cancer Cell Lines

Fluorescence quantitative PCR was used in identifying renal cancer cell lines (ACHN, 796-p, 786-O, and Caki02) and standard renal hollow epithelial cells (HK-2), and the effects of S100A16 on the onset and progression of renal growth were investigated. Similar to ordinary renal tubular epithelial cells (HK-2), S100A16 was strongly expressed in renal cancer cell lines, with the 796-P cell line exhibited the highest expression level (Figure 8(a)). 796-P cells were transfected with an S100A16 knockdown vector (shRNA-S100A16) and a control group (shRNA-control), and the unique regulatory role of S100A16 in renal cancer cells was characterized. Fluorescence quantitative PCR results demonstrated that the transfection of shRNA-S100A16 substantially inhibited the expression level of S100A16.0 mRNA in renal cancer 796-P cells compared with the control group (shRNA-control; Figure 8(b)). Western blot analysis results revealed that transfection of shRNA-S100A16 substantially inhibited the expression level of S100A16 protein in renal cancer 796-P cells compared with the control group (shRNA-control; Figure 8(c)).

Additionally, the effects of S100A16 on the proliferation and migration of renal cancer cells were investigated using a CCK-8 detection assay. The findings indicated that related control cluster (shRNA-control), the S100A16.0 knockdown vector (shRNA-S100A16), can be transfected, significantly inhibiting the capacity of kidney carcinoma cells to proliferate (Figure 9(a)). The findings of the clone creation experiment demonstrated that, compared with the control group (shRNA-control), the transfection of the S100A16.0 knockdown vector (shRNA-S100A16) greatly inhibited the capacity of kidney cancer cells to generate clones (Figure 9(b)). The findings of the Transwell cell migration experiment demonstrated, compared with the control group (shRNA-control), the transfection of the S100A16.0 knockdown vector (shRNA-S100A16) substantially inhibited renal cancer cell movement (Figure 9(c)).

We performed an angiogenesis experiment to determine the effect of knocking down S100A16 expression on the angiogenesis of renal carcinoma cells. Compared with the control group (shRNA-control), the transfection of the S100A16 knockdown vector (shRNA-S100A16) dramatically inhibited angiogenesis in the renal cancer cells (Figure 10(a)). Compared with the control group (shRNA-control), the transfection of the S100A16.0 knockdown vector (shRNA-S100A16) dramatically suppressed the production of VEGF, VEGFR2, and phosphorylated AKT (p-Akt) in renal cancer cells but had no impact on the expression of total Akt (Figure 10(b)).

## 4. Discussion

In urological cancer, RCC remains the second highest cause of mortality [17]. In 2018, an estimated total of 403,000.0 cases of renal cell carcinoma were reported, resulting in 175 thousand fatalities [18]. In China, 68,300.0 cases and 25,600 deaths from renal cell carcinoma were recorded in 2014. The overall 5-year survival rate for patients with RCC has increased from 50% to 74% in the last three decades. This increase is mostly attributed to the rising number of early-stage RCC and the increased use of medical imaging [19, 20]. Therapy for advanced or metastatic RCC remains limited partly because of the high recurrence rates and distant metastases despite advances in early identification methods. Clarifying the mechanism behind the formation and progression of RCC is crucial to the identification of relevant biomarkers and development of novel treatment methods.

Developments in sequencing and omics technologies have facilitated the exploration of diagnostic and therapeutic targets [21]. In this work, we used a combination of bioinformatics analysis and in vitro tests to investigate the function of S100A16 in the formation and evolution of RCC and the potential mode of action. In the TCGA database, we discovered that S100A16 expression was elevated in RCC, and individuals with RCC and high S100A16 expression levels had lower OS, DSS, and PFI than those with low S100A16 expression levels. In addition, we built a nomogram by evaluating the association between S100A16 and the clinical parameters of the patients to enhance the clinical value of the prediction. The results of additional data analysis in the TIMER database and the correlation with immune checkpoint-related molecules CTLA-4, CD274, and PDCD1 indicated that the expression of S100A16 is significantly associated with immune infiltration and S100A16 plays a crucial role in promoting immune escape of tumor cells in the RCC tumor microenvironment. Next, we investigated the relationship between S100A16 and the existing RCC-targeted pharmacological therapy's target molecules. S100A16 was strongly associated with AXL, EGFR, FLT3, KIT, MET, NTRK2, RET, TEK, and VEGFA. These data may serve as references for selecting targeted medications. Currently, global clinical trials, such as the CLEAR study-KEYNOTE-581 study, demonstrated that the phase III randomized controlled study of pembrolizumab combined with lenvatinib as the first-line treatment of advanced RCC met the primary study endpoint, and efficacy was significantly enhanced [22]. CheckMate 9er study: first-line combination therapy with nivolumab plus cabozantinib in advanced RCC, in which the combination was compared with sunitinib, Orr 54.6% vs 28.4%; median PFS 17 months vs 8.3 months, and median OS NR vs. 29.5 months. The results demonstrated that immunological combination targeted treatment was considerably superior to sunitinib [23]. Adjuvant TKI treatment did not enhance OS following nephrectomy in neoadjuvant and adjuvant therapy for renal cell cancer according to the 2022 EAU recommendations. Pembrolizumab usage adjuvant to nephrectomy increased progression-free survival in patients with RCC at high risk. Adjuvant pembrolizumab enhanced disease-free survival in selected intermediate- or high-risk individuals or in M1 patients with no indication of illness in a randomized controlled study. Non-ccmRCC is resistant to mTOR inhibitors and VEGF-targeted treatment in metastatic RCC. Sunitinib had no discernible effect on oncologic outcomes when compared to everolimus. In non-cc-mRCC, sunitinib increased progression-free survival (PFS), versus everolimus, in phase II studies and a comprehensive analysis of patient subgroups. Compared with sunitinib, savolitinib increased PFS in patients with MET-driven advanced pRCC. Pembrolizumab in a single-arm trial in the pRCC subgroup led to a shift in category 2a evidence for long-term median OS [24, 25]. Therefore, immunotherapy coupled with targeted therapy may be a more effective therapeutic choice for RCC that has relapsed or spread. In addition, the molecule S100A16 investigated in this study is associated not only with the immune infiltration of RCC but also with the target molecule, indicating that our research has some therapeutic utility.

We predicted the signaling pathway by using KEGG of GSEA. We discovered that S100A16 may influence the biological processes of RCC by engaging in the VEGF/VEGFR2 signaling pathway, P53 alterations, cell cycle, and PI3K-Akt signaling pathway, therefore altering the prognosis of RCC. By modulating the PI3K/AKT signaling pathway, S100A16 may boost the proliferation, migration, and tumor angiogenesis of HeLa cells [26]. In human prostate cancer, S100A16 increases cell proliferation and metastasis through the AKT and ERK cell signaling pathways [15]. The calcium-binding protein S100A16 may contribute to the poor prognosis of RCC by boosting renal cell carcinoma development and angiogenesis through the VEGF/VEGFR2 signaling pathway. Consequently, we conducted cytological tests to confirm the presence of S100A16 in RCC. We first compared the expression levels of S100A16 in normal renal tubular epithelial cells (HK-2) and renal cancer cell lines (ACHN, 796-p, 786-O, and Caki02). We discovered that the expression of S100A16 was elevated in all four RCC cell lines, and the 796-P cell line had the highest expression. Consequently, 796-P was used in subsequent cytological investigations. The findings suggested that the suppression of S100A16 inhibits the proliferation, clone formation, and migration of renal cancer cells. Moreover, the angiogenesis studies demonstrated that the suppression of S100A16 may reduce the expression levels of VEGF, VEGFR2, and p-Akt in renal cancer cells, consequently diminishing their angiogenesis capacities. Previous research [27] has shown that diosgenin inhibits AKT phosphorylation and promotes apoptosis in human kidney carcinoma ACHN cells by activating P53. FoxO transcription factor enhances AKT Ser473 phosphorylation and renal tumor development in response to PI3K-AKT pathway suppression [28]. SGK2 enhances the development of renal carcinoma by increasing ERK1/2 and AKT phosphorylation [29]. The significance of p-Akt in the biological processes of RCC is supported by these findings and our cytological research.

## 5. Conclusion

In conclusion, many lines of evidence support the significance of S100A16 in RCC formation and its potential as a biomarker for the progression of RCC illness. Interfering with S100A16 may enhance the development and angiogenesis of RCC through the VEGF/VEGFR2 signaling pathway, hence altering the dismal prognosis of RCC. These results indicate a possible target for the development of anticancer therapy against RCC.

## Figures and Tables

**Figure 1:** Elevated S100A16 expression in RCC. (a) S100A16 expression in renal clear cell carcinoma. (b) Expression of S100A16 in RCC unpaired tissues (tumor 539-normal 72). (c) S100A16 expression in paired RCC and normal tissue (tumor 72 -normal 72). (d) S100A16 ROC analysis demonstrated ability to distinguish between tumor and normal tissues. ^*∗*^*p* < 0.05, ^*∗∗*^*p* < 0.01, ^*∗∗∗*^*p* < 0.001. Relationship between S100A16 in TCGA database and clinical data of RCC.

**Figure 2:** Correlation between S100A16 and clinical data of patients with RCC. ^*∗*^*p* < 0.05, ^*∗∗*^*p* < 0.01, ^*∗∗∗*^*p* < 0.001.

**Figure 3:** Prognoses of S100A16 and patients with RCC in the TCGA database. (a). Low S100A16 expression was associated with improved OS, DSS, and PFI in the patients. (b). Stratified subgroup analysis revealed that the prognosis for individuals with low S100A16 expression was more favorable.

**Figure 4:** Nomogram and calibration plot. (a) Nomogram used to predict the 1-, 3-, and 5-year OS rates of patients with RCC. (b) Calibration plot of the nomogram utilized in predicting OS probability. Correlation between S100A16 and immune cells in the TIMER database.

**Figure 5:** Correlation between s100a16 and immune cells in the TIMER database. (a) S100a16 was positively correlated with the infiltration of most immune cells in the TIMER database; (b) S100a16 expression was significantly associated with immune cell infiltration in RCC; (c) scatter plot of the correlation between s100a16 expression and CTLA-4, CD274, and PDCD1 in RCC.

**Figure 6:** Correlation between S100A16 and pharmacological targets for molecular targeted therapies in the TCGA database. Prediction of KEGG signaling pathway based on GSEA.

**Figure 7:** Four potentially relevant pathways with statistical significance.

**Figure 8:** In renal cancer cell lines, S100A16 was significantly expressed. (a) Detection of S100A16 expression in renal carcinoma cell lines through real-time PCR. (b, c) Fluorescence quantitative PCR detection of S100A16.0 in renal cancer cells after transfection and suppression of S100A16 vector mRNA and protein levels, ^*∗∗*^*p* < 0.01. Effects of the knockdown of S100A16 on the proliferation and migration of renal cancer cells.

**Figure 9:** Effects of S100A16 on the proliferation and migration of renal cancer cells. (a) CCK-8 was used in detecting the effect of S100A16 knockdown on the proliferation of renal cancer cells, and (b) clone creation was performed for the analysis of the inhibiting effects of S100A16 on renal cancer cell movement. Influence on cell clonogenicity, ^*∗∗*^*p* < 0.01. (c) The effect of S100A16 knockdown on the migration of renal cancer cells, ^*∗∗*^*p* < 0.01. Effects of knockdown of S100A16 on angiogenesis in renal cancer cells.

**Figure 10:** Impact of S100A16 knockdown on angiogenesis in renal cancer cells. (a) Angiogenesis test for identifying the impact of S100A16 knockdown on angiogenesis in renal cancer cells. (b) Western blot for identifying the main angiogenesis protein after S100A16 knockdown ^*∗∗*^*p* < 0.01, ^*∗*^*p* < 0.05, ^*∗∗∗*^*p* < 0.01.

## Data Availability

The data are available from the corresponding author upon request via e-mail (15857256165@163.com).
